The article "LncRNA SNHG14 contributes to the progression of NSCLC through miR‐206/G6PD pathway" was retracted in 2025. Reasons: errors in the materials; unreliable results or conclusions.

# LncRNA SNHG14 contributes to the progression of NSCLC through miR‐206/G6PD pathway

**DOI:** 10.1111/1759-7714.13374

**Published:** 2020-03-09

**Authors:** Lin Zhao, Xiaodong Zhang, Yantong Shi, Tianlu Teng

**Affiliations:** ^1^ Department of Respiratory Medicine Affiliated Rizhao People's Hospital of Jining Medical University Rizhao China; ^2^ Departmentof Clinical Laboratory, Rizhao Center for Disease Control and Prevention Rizhao China; ^3^ Department of Respiratory Medicine, Beijing Chest Hospital, Capital Medical University Beijing China

**Keywords:** G6PD, lncRNA SNHG14, miR‐206, NSCLC

## Abstract

**Background:**

Previous studies have shown that the dysregulation of lncRNAs participates in non‐small cell lung cancer (NSCLC) development. The purpose of this study was to research the biological function of lncRNA SNHG14 and its molecular mechanism in NSCLC progression.

**Methods:**

RT‐PCR was applied for investigating the expression of SNHG14, miR‐206 and G6PD. The progression of NSCLC was detected by CCK‐8, Transwell and western blot assays. The targets of SNHG14 and miR‐206 were measured by dual‐luciferase reporter assay.

**Results:**

We found a higher expression of SNHG14 in NSCLC and upregulation of SNHG14 contributed to NSCLC cell proliferation, invasion and migration. However, knockdown of SNHG14 showed the opposite effect on the progression of NSCLC. Specifically, SNHG14 negatively regulated miR‐206 expression by binding with it directly. Furthermore, G6PD served as the target of miR‐206. Rescue experiments showed that SNHG14 promoted G6PD expression by inhibiting miR‐206.

**Conclusions:**

LncRNA SNHG14 contributed to NSCLC progression through miR‐206/G6PD axis, providing novel clues for understanding the mechanism of NSCLC.

## Introduction

Lung cancer is a malignant tumor with the highest morbidity and mortality in China, which seriously threatens the life and health of people.^1^, ^2^ More than 85% of lung cancer patients are diagnosed with non‐small cell lung cancer (NSCLC).^3^ In the past 50 years, the incidence and mortality of lung cancer has been reported to have increased significantly, accounting for the first in all malignant tumors, especially in men.^4^ Currently, researchers have spared no efforts to explore the pathogenesis of lung cancer in order to apply it to clinical treatment as soon as possible.^5^, ^6^ However, effective interventions and procedures for NSCLC have so far been rare. Therefore, searching for new therapeutic targets is very important.

LncRNAs have been reported to participate in the progression of various types of tumors,^7^, ^8^, ^9^ including lung cancer.^10^, ^11^ For example, Yu *et al*. found that lncRNA FBXL19‐AS1 was highly expressed in NSCLC and its high expression enhanced cell proliferation and metastasis.^12^ Zheng and colleagues revealed that lncRNA HOXA‐AS2 played a facilitating role in NSCLC metastasis.^13^ The role of lncRNA NORAD in NSCLC was discovered by Chen *et al*. in promoting the development of lung cancer.^14^ However, the role of lncRNA SNHG14 in lung cancer remains unclear. LncRNA SNHG14, alternatively named UBE3AATS, has been reported to be involved in the development of tumors, including ovarian cancer, bladder and cervical cancer.^15^, ^16^, ^17^ Here, we explored the role of lncRNA SNHG14 in NSCLC progression, and investigated whether SNHG14 was expressed abnormally in NSCLC. Moreover, SNHG14 expression was increased or decreased in NSCLC cells to investigate the biological function of SNHG14 in NSCLC cell proliferation, invasion and migration. Additionally, a previous study showed that SNHG14 promoted cervical cancer progression by regulating miR‐206,^18^ and Cui *et al*. found that miR‐206 hindered cervical cancer cell proliferation by targeting G6PD.^19^ Thus, in our study, we explored whether SNHG14 could modulate miR‐206/G6PD axis to better understand the mechanism of SNHG14 in the regulation of the progression of NSCLC.

The article "LncRNA SNHG14 contributes to the progression of NSCLC through miR‐206/G6PD pathway" was retracted in 2025. Reasons: errors in the materials; unreliable results or conclusions.

Here, we investigated both the functional role and molecular mechanism of SNHG14 in the modulation of NSCLC progression, with the aim of providing a new diagnostic predictor and a valuable therapeutic target for NSCLC.

## Methods

### Study subjects

A total of 74 paired NSCLC and normal tissue specimens were collected from NSCLC patients. These did not include patients who had received any treatment before surgery. The tissues were scored at −80°C for further use. Written informed consents were provided by all participants and the ethics committee of the Affiliated Rizhao People's Hospital of Jining Medical University approved this study.

### Cell culture and cell transfection

Normal human bronchial epithelial 16HBE cells and two NSCLC cell lines (A549 and SK‐MES‐1) provided by ATCC were cultured in RPMI 1640 medium containing 10% FBS and maintained at 37°C with 5% CO_2_ atmosphere.

MiR‐206 mimic or inhibitor, SNHG14 siRNA or vector and their corresponding controls were provided by GenePharma (Shanghai, China). They were delivered to A549 and SK‐MES‐1 cells with the aid of Lipofectamine 2000 reagent (Invitrogen). After transfection for 48 hours, the cells were collected for further analysis.

### RT‐PCR

TRizol reagent was applied for extracting total RNA from prepared tissues or cells. A NanoDrop 2000 spectrophotometer (Thermo, MA, USA) was used for measuring the RNA concentration and quality. PrimeScript RT reagent Kit (TaKaRa) and OneStep PrimeScript miRNA cDNA Synthesis Kit (Qiagen, CA, USA) were used to perform reverse transcription in lncRNA and miRNA quantification, respectively. SYBR Premix Ex Taq II kit (Takara) was used to determine qPCR analysis. GAPDH and U6 were applied for normalization of lncRNA and miRNA, respectively. The expression of tested genes was calculated by 2‐ΔΔCt method. The primers sequences used are listed in Table 1.

The article "LncRNA SNHG14 contributes to the progression of NSCLC through miR‐206/G6PD pathway" was retracted in 2025. Reasons: errors in the materials; unreliable results or conclusions.

### Western blot

RIPA buffer containing protease inhibitors was applied for preparing cell lysates. After proteins were separated by SDS‐PAGE, followed by transfer to NC membranes, they were incubated with nonfat milk for 1 hour. Primary antibodies were subsequently incubated overnight at 4°C and then secondary antibodies for 1 hour. The primary antibodies used in this study were anti‐G6PD antibody and anti‐GAPDH antibody.

### CCK‐8 assay

A CCK‐8 Kit was used to assay the altered cell viability after different transfections. After transfection with miR‐206 mimic, SNHG14 siRNA or vector and their corresponding controls, NSCLC cells were seeded into 48‐well plates and cultured for one, two, three, and four days. The cells were then treated with CCK‐8 solution for another 2 hours. Finally, a spectrophotometer (Thermo, MA, USA) was applied to measure the optical density at 450 nm.

### Transwell assays

Transwell chambers precoated with or without Matrigel were used to detect cell invasion and migration. Two NSCLC cell lines with different transfections after transfection with miR‐206 mimic, SNHG14 siRNA or vector and their corresponding controls, were added inside the chamber. Next, DMEM medium containing 10% FBS was seeded into a 24‐well plate and placed into the transwell chamber. After incubation for 24 hours, the invaded or migrated cells was fixed, stained and counted.

### Luciferase reporter assay

The amplified wild‐ or mutant type of SNHG14 3′UTR (SNHG14 3′UTR‐WT, ‐MUT) was cloned into the pGL3‐reporter vector. With the aid of Lipofectamine 2000 reagent, miR‐206 mimic or inhibitor and SNHG14‐WT or ‐MUT were cotransfected into A549 cells. At 48 hours post‐transfection, luciferase activity was detected.

### Statistical analysis

The values were analyzed by SPSS 22.0 software and presented as mean ± SD. *P*‐value significance between the two groups was compared with a Student's *t*‐test. Tukey's post hoc test was applied for comparing the significance between multiple groups. *P* < 0.05 was considered as statistically significant.

## Results

### SNHG14 was increased in NSCLC

To detect the role of lncRNA SNHG14' in NSCLC development, the expression level of SNHG14 was first measured in NSCLC tissues and cells. As a result, the expression level of SNHG14 was dramatically increased in NSCLC tissues compared with nontumor tissues (Fig 1a). Moreover, similar results were found in NSCLC cells. In NSCLC cells, SNHG14 expression was higher relative to that in normal cells (Fig 1b). These data suggested that high expression of SNHG14 might play a critical role in NSCLC development.

The article "LncRNA SNHG14 contributes to the progression of NSCLC through miR‐206/G6PD pathway" was retracted in 2025. Reasons: errors in the materials; unreliable results or conclusions.

**Figure 1:** SNHG14 was increased in NSCLC. (**a**) There was a higher expression of SNHG14 in NSCLC tissues than in nontumor tissues. (**b**) Increased expression of SNHG14 in NSCLC cells (A549 and SK‐MES‐1 cells) in comparison with that in normal 16HBE cells. *P < 0.05.

**Table 1:** Primer sequences for RT‐qPCR

Primer	Sequence
SNHG14	
Forward	5′‐GGGTGTTTACGTAGACCAGAACC‐3′
Reverse	5′‐CTTCCAAAAGCCTTCTGCCTTAG‐3′
miR‐206	
Forward	5′‐CCAAAGCGGAGTCTCGCAT‐3′
Reverse	5′‐GCCTAGCATCTTGCTTAGCTC‐3′
U6	
Forward	5′‐GCTTCGGCAGCACATATACTAAAAT‐3′
Reverse	5′‐CGCTTCACGAATTTGCGTGTCAT‐3′
G6PD	
Forward	5′‐TGCCTTCCATCAGTCGGATACAC‐3′
Reverse	5′‐TGGTGGGGTAGATCTTCTTCTTGG‐3′
GAPDH	
Forward	5′‐CCAAAATCAGATGGGGCAATGCTGG‐3′
Reverse	5′‐TGATGGCATGGACTGTGGTCATTCA‐3′

G6PD, Glucose‐6‐phosphate dehydrogenase; GAPDH, glyceraldehyde‐3‐phosphate dehydrogenase; U6, small nuclear RNA, snRNA.

### SNHG14 modulated NSCLC progression

Next, we examined the effect of SNHG14 on NSCLC progression. Two cancer cells were transfected with SNHG14 siRNA or vector to knockdown or overexpress SNHG14. As show2a, the high knockdown or overexpression efficiency was determined by RT‐PCR. CCK‐8 assay results showed that decreasing SNHG14 repressed cells, whereas increasing SNHG14 promoted the viability of NSCLC cells (Fig 2b,c). In addition, the findings of transwell migration assay revealed that silencing SNHG14 suppressed cells, while upregulation SNHG14 enhanced the number of migrated cells in both NSCLC cells (Fig 2d). Moreover, the number of invaded cells was also hindered by SNHG14 siRNA, whereas it was facilitated by SNHG14 vector (Fig 2e). These findings indicated that SNHG14 contributes to NSCLC progression.

**Figure 2:** SNHG14 modulated NSCLC progression. (**a**) Measurement of SNHG14 expression in two NSCLC cells after overexpression or silencing SNHG14. () NC siRNA, () SNHG14 siRNA, () NC vector and () SNHG14 vector. (**b**) Cell viability. A549 () SNHG14 vector, () NC vector, () SNHG14 siRNA and () NC siRNA. (**c**) Cell viability. SK‐MES‐1 () SNHG14 vector, () NC vector, () SNHG14 siRNA and () NC siRNA. (**d**) Cell migration. () NC siRNA, () SNHG14 siRNA, () NC vector and () SNHG14 vector. (**e**) Cell invasion. () NC siRNA, () SNHG14 siRNA, () NC vector and () SNHG14 vector. *P < 0.05, **P < 0.01.

The article "LncRNA SNHG14 contributes to the progression of NSCLC through miR‐206/G6PD pathway" was retracted in 2025. Reasons: errors in the materials; unreliable results or conclusions.

### SNHG14 acts as a sponge for miR‐206 in NSCLC cells

By using the bioinformatic tool starBase, miR‐206 was predicted as the target of SNHG14 (Fig 3a). Dual luciferase reporter assay was then performed to validate the direct binding between miR‐206 and SNHG14. As show3b,c, the luciferase activity of SNHG14‐WT was decreased in the A549 and SK‐MES‐1 cells treated with miR‐206 mimic in comparison with the control, whereas it increased when treated with miR‐206 inhibitor. However, the luciferase activity of SNHG14‐MUT showed no change when treated with transfection of miR‐206 mimic, miR‐206 inhibitor, con mimic, con inhibitor. We then tested miR‐206 expression in NSCLC tissues. As shown in Fig 3d, it was decreased in NSCLC tissues relative to normal control. Because its expression was opposite to SNHG14 expression, we investigated whether miR‐206 was modulated by SNHG14. The findings revealed that re‐expression of SNHG14 were inhibited, while knockdown of SNHG14 facilitated miR‐206 mRNA expression (Fig 3e). These data showed that miR‐206 was the target of SNHG14 in NSCLC.

**Figure 3:** SNHG14 acted as a sponge for miR‐206 in NSCLC cells. (**a**) The prediction binding sites of SNHG14 and miR‐206 are shown. (**b**, **c**) The luciferase activity detected in A549 and SK‐MES‐1 cells with a different transfection of miR‐206 mimic, miR‐206 inhibitor, con mimic, con inhibitor. () con mimic, () miR‐206 mimic, () con inhibitor and () miR‐206 inhibitor. () con mimic, () miR‐206 mimic, () con inhibitor and () miR‐206 inhibitor. (**d**) The expression level of miR‐206 measured in NSCLC tissues. (**e**) The mRNA level of miR‐206 tested in the two NSCLC cells with different transfections of NC siRNA, SNHG14 siRNA, NC vector and SNHG14 vector. () NC siRNA, () SNHG14 siRNA, () NC vector and () SNHG14 vector. *P < 0.05, **P < 0.01.

### SNHG14 regulated NSCLC development by targeting miR‐206

Next, we explored miR‐206 effect on SNHG14 in modulating NSCLC development. Two cancer cells were treated with SNHG14 siRNA or vector, combined with miR‐206 mimic. The cell viability was decreased in the SNHG14 siRNA group compared with the control group, and significantly decreased in the SNHG14 siRNA+miR‐206 mimic group in comparison with the SNHG14 siRNA group (Fig 4a). However, the cell viability was increased by the SNHG14 vector, while inhibited by the miR‐206 mimic (Fig 4b). Moreover, transwell migration assay results showed that the miR‐206 mimic further promoted the inhibitory effect of SNHG14 siRNA on cell migration (Fig 4c), and overturned the promoting effect of SNHG14 vector on cell migration (Fig 4d). More importantly, similar trends of cell invasion and cell migration were observed in Fig 4e,f. In summary, these findings demonstrated that SNHG14 modulated NSCLC progression by targeting miR‐206.

The article "LncRNA SNHG14 contributes to the progression of NSCLC through miR‐206/G6PD pathway" was retracted in 2025. Reasons: errors in the materials; unreliable results or conclusions.

**Figure 4:** SNHG14 modulated NSCLC progression by targeting miR‐206. Two NSCLC cells were transfected with SNHG14 siRNA or vector, combined with miR‐206 mimic. (**a and b**) Cell viability in NSCLC cells after being treated with different transfections SNHG14 siRNA or vector, combined with miR‐206 mimic. () SNHG14 siRNA+miR‐206 mimic, () SNHG14 siRNA and () control. () SNHG14 siRNA+miR‐206 mimic, () SNHG14 siRNA and () control. (**c and d**) Cell invasion and (**e** and **f**) cell migration in the two NSCLC cells with different transfections of SNHG14 siRNA or vector, combined with miR‐206 mimic. *P < 0.05, **P < 0.01.

### G6PD was the target of miR‐206

TargetScan was applied for predicting the potential targets of miR‐206 and G6PD was identified as the possible target (Fig 5a). To further verify the predicted target relationship, dual luciferase reporter assay was applied. As seen in Fig 5b,c, miR‐206 mimic significantly reduced the luciferase activity of G6PD 3′UTR‐WT, but not G6PD 3′UTR‐MuT. Moreover, we detected G6PD expression was affected by miR‐206. Results showed that the mRNA and protein level of G6PD was significantly decreased by overexpression of miR‐206, while increased by inhibiting miR‐206 (Fig 5d,e). These findings suggested that G6PD served as miR‐206′ direct target.

**Figure 5:** G6PD served as the target of miR‐101 in NSCLC cells. (**a**) MiR‐206 and G6PD are the binding sites. (**b**, **c**) The luciferase activity of G6PD 3′UTR‐WT or ‐MUT in A549 and SK‐MES‐1 cells after being treated with different transfections of miR‐206 mimic, miR‐206 inhibitor, con mimic, con inhibitor. A549 () con mimic, () miR‐206 mimic, () con inhibitor and () miR‐206 inhibitor. SK‐MES‐1 () con mimic, () miR‐206 mimic, () con inhibitor and () miR‐206 inhibitor. (**d**, **e**) The protein level and mRNA level of G6PD tested in the two NSCLC cells with different transfections. () con mimic, () miR‐206 mimic, () con inhibitor and () miR‐206 inhibitor. *P < 0.05, **P < 0.01.

### G6PD served as a downstream target of SNHG14 in NSCLC cells

We then explored whether G6PD was modulated by SNHG14 via miR‐206. As show6a, SNHG14 upregulation facilitated G6PD mRNA and protein expression and was then repressed when combined with the miR‐206 mimic. However, knockdown of SNHG14 suppressed G6PD expression, while simultaneously with overexpression of miR‐206 further inhibited G6PD expression (Fig 6b). In addition, in NSCLC tissues, the relationship between G6PD expression and SNHG14 expression was positive (Fig 6c), but the correlation of G6PD with miR‐206 expression was negative (Fig 6d). This confirms that SNHG14 enhanced G6PD expression via hindering miR‐206 expression in NSCLC.

The article "LncRNA SNHG14 contributes to the progression of NSCLC through miR‐206/G6PD pathway" was retracted in 2025. Reasons: errors in the materials; unreliable results or conclusions.

**Figure 6:** G6PD served as the downstream target of SNHG14 in NSCLC. (**a**) G6PD mRNA. () Control, () SNHG14 vector and () SNHG14 vector+miR‐206 mimic. (**b**) G6PD protein level detected in the two NSCLC cells with different transfections of SNHG14 vector and miR‐206 mimic. () Control, () SNHG14 siRNA and () SNHG14 siRNA+miR‐206 mimic. (**c**) The relationship between G6PD and SNHG14 expression. (**d**) The relationship between G6PD and miR‐206 expression. *P < 0.05, **P < 0.01.

## Discussion

In the present study, we showed that SNHG14 was highly expressed in NSCLC tissues and cells. Overexpression of SNHG14 contributed to cell proliferation, invasion and migration. However, knockdown of SNHG14 inhibited NSCLC progression. More importantly, miR‐206 was verified as the downstream effector of SNHG14 and G6PD was the direct target of miR‐206. Moreover, we proved that SNHG14 could facilitate G6PD expression by impeding miR‐206. Collectively, we demonstrated that SNHG14 contributed to NSCLC progression by regulating miR‐206/G6PD axis.

There is increasing evidence that lncRNAs are related to the development of various tumors. Previous studies have showed that lncRNA SNHG14 promoted clear cell renal cell carcinoma migration and invasion as an oncogene.^20^ Also, Liu *et al*. revealed that SNHG14 facilitated the development of gastric cancer.^21^ Dong *et al*. showed that SNHG14 promotes trastuzumab chemoresistance in breast cancer.^22^ Similar results were found in our study. We reported that lncRNA SNHG14 was highly expressed in NSCLC tissues. Overexpression lncRNA SNHG14 facilitated, while silence lncRNA SNHG14 inhibited NSCLC proliferation, invasion and migration. Briefly, lncRNA SNHG14 revealed the promotion effect on the development of NSCLC.

LncRNAs have been reported to sponge miRNAs to modulate the derepression of miRNA targets, consequently regulating the progress of different diseases.^23^ For example, Li and colleagues showed that SNHG14 acted as sponge for miR‐219 and miR‐125 in facilitating ovarian cancer viability and metastasis.^16^, ^24^ Xie *et al*. found that miR‐193a served as the target of SNHG14 in promoting breast cancer cell proliferation and invasion.^25^ More importantly, SNHG14 conferred the gefitinib resistance via miR‐206/ABCB1 axis in NSCLC.^26^ Here, for the first time we showed that SNHG14 served as a sponge for miR‐206 in promoting lung cancer cell viability, invasion and migration.

As already determined, miRNAs regulate tumors development by targeting their mRNAs through binding to 3′UTR. In lung cancer, miR‐206 is reported to target several mRNA genes. For instance, MET function as the target of miR‐206 in suppressing lung cancer progression.^27^ Moreover, Ren *et al*. showed that miR‐206 showed suppression effect on colorectal cancer via targeting FMNL2.^28^ Zhang *et al*. reported that SOX9 took part in NSCLC progression as the target of miR‐206.^29^ In this study, we determined G6PD as the target of miR‐206 in NSCLC. Specifically, we proved that SNHG14 positively regulated G6PD expression by sponging miR‐206 in NSCLC.

The article "LncRNA SNHG14 contributes to the progression of NSCLC through miR‐206/G6PD pathway" was retracted in 2025. Reasons: errors in the materials; unreliable results or conclusions.

In summary, we conclude that SNHG14 plays a role in NSCLC. The promotion role of SNHG14 in NSCLC progression could be inhibited by miR‐206. SNHG14 enhanced G6PD expression by suppressing miR‐206. Our results provide evidence that SNHG14/miR‐206/G6PD axis regulated the development of NSCLC. Therefore, SNHG14 might serve as a promising therapeutic target for NSCLC.

## Disclosure

No authors report any conflict of interest.
